RETRACTED

# Prenatal Cocaine Exposure Upregulates BDNF-TrkB Signaling

**DOI:** 10.1371/journal.pone.0160585

**Published:** 2016-08-05

**Authors:** Andres Stucky, Kalindi P. Bakshi, Eitan Friedman, Hoau-Yan Wang

**Affiliations:** 1 Departments of Physiology, Pharmacology and Neuroscience, School of Medicine at CCNY, The City University of New York, New York, New York, 10031, United States of America; 2 Department of Biology, Neuroscience Program, Graduate School of The City University of New York, New York, New York, 10061, United States of America; University of South Carolina School of Medicine, UNITED STATES

## Abstract

Prenatal cocaine exposure causes profound changes in neurobehavior as well as synaptic function and structure with compromised glutamatergic transmission. Since synaptic health and glutamatergic activity are tightly regulated by brain-derived neurotrophic factor (BDNF) signaling through its cognate tyrosine receptor kinase B (TrkB), we hypothesized that prenatal cocaine exposure alters BDNF-TrkB signaling during brain development. Here we show prenatal cocaine exposure enhances BDNF-TrkB signaling in hippocampus and prefrontal cortex (PFCX) of 21-day-old rats without affecting the expression levels of TrkB, P75^NTR^, signaling molecules, NMDA receptor—NR1 subunit as well as proBDNF and BDNF. Prenatal cocaine exposure reduces activity-dependent proBDNF and BDNF release and elevates BDNF affinity for TrkB leading to increased tyrosine-phosphorylated TrkB, heightened Phospholipase C-γ1 and N-Shc/Shc recruitment and higher downstream PI3K and ERK activation in response to *ex vivo* BDNF. The augmented BDNF-TrkB signaling is accompanied by increases in association between activated TrkB and NMDARs. These data suggest that cocaine exposure during gestation upregulates BDNF-TrkB signaling and its interaction with NMDARs by increasing BDNF affinity, perhaps in an attempt to restore the diminished excitatory neurotransmission.

## Introduction

Studies in both humans and animal, have shown that prenatal cocaine exposure can negatively affect attention, motor, and language skills, as well as associative and discrimination learning, all of which involve excitatory synapses [1–4]. Cocaine exposure during gestation causes impaired synaptic plasticity[5] that may be related to developmental delays in the excitatory glutamatergic systems [6]. There is also evidence indicating prenatal cocaine exposure leads to increased spine density in the cortical and subcortical regions [7] as well as hypertrophic dendritic outgrowth with atypical, tortuous dendritic profile [8]. Although the latter change in dendritic structure has been attributed to uncoupling of the dopamine D_1_ receptor from its associated Gs/olf protein, BDNF-TrkB signaling is one of the prominent upstream modulators of the glutamatergic function and dendritic health in brain areas such as neocortex and hippocampus [9–11]. It is therefore highly conceivable the defects in glutamatergic neurotransmission and abnormal dendritic morphology found in prenatal cocaine exposed brains are partly caused by altered BDNF-TrkB signaling.

RETRACTED

In response to BDNF, TrkB is tyrosine phosphorylated (activated) by its intrinsic tyrosine kinase that leads to recruitment of phospholipase C-γ1 and increases downstream ERK2 and PI3K activities through the association of adaptor proteins such as Shc and N-Shc with phosphotyrosine residues on activated TrkB [12]. Functionally, TrkB activation by BNDF increases expression of immediate early response genes relevant to synaptic plasticity and promotes pleiotropic effects on various cells [13, 14]. During brain development and maturation, BDNF-TrkB signaling is essential for proper neuronal migration [15, 16] as well as the establishment and survival of glutamatergic connections [17]. Through activation of TrkB, BDNF upregulates glutamatergic transmission and N-Methyl-D-Aspartate receptor (NMDAR) function, which in turn promotes phosphorylation of the NMDA receptor channels. Autophosphorylation of the kinase domain of TrkB activates signaling cascades that promote cell growth and survival [18] and the maintenance of active synaptic connections [19].

BDNF is synthesized as a precursor protein (proBDNF) in the endoplasmic reticulum. Following cleavage of the signal peptide, the resultant proBDNF is then transported to the Golgi for sorting into either constitutive or regulated secretory vesicles for spontaneous and activity-regulated release. Although the efficiency of intracellular cleavage remains controversial [20] and likely varies among neuronal cell types, findings suggest that exposure to cocaine during early development can modify synaptic plasticity at excitatory synapses, causing long-lasting alterations in brain activity and function leading to altered activity-dependent proBDNF/BDNF release. In support of this possibility, our earlier data indicate that cocaine exposure *in utero* attenuates AMPAR-mediated LTD without affecting basal transmission [21]. Since BDNF-TrkB regulates glutamatergic synaptic transmission, we investigated whether prenatal cocaine affects BDNF/TrkB signaling and the underlying mechanism responsible for such changes. Our results show that prenatal cocaine exposure decreases activity-dependent BDNF and proBDNF release and leads to increased BDNF affinity for TrkB receptors and enhanced efficiency of the BDNF-TrkB signaling.

RETRACTED

## Materials and Methods

### Materials and chemicals

Recombinant human BDNF (rhBDNF), Leupeptin, aprotinin, phenylmethylsulfonyl fluoride (PMSF), pepstatin A, soybean trypsin inhibitor, NaF, sodium vanadate, β-glycerophosphate, 2-mercaptoethanol, NMDA, glycine, Tween-20, NP-40 and digitonin were from Sigma-Aldrich (Saint Louis, MO). Anti-phosphotyrosine (SC-508), TrkB (SC-119) -ERK2 (SC-154, SC-81457), -pT^202^/ pY^204^-ERK (SC-136521), -pS^473^Akt (SC- 7985-R), -Akt1 (SC-65487), -Akt1/2/3 (SC-8312), -phospholipase C-γ1 (SC-7290), -Shc (SC-967), -N-Shc (SC-28833) -NR1 (SC-9058), -actin (SC-7210), -β-actin (SC-47778), -p75^NTR^ (SC-6189, SC-55467), -TRAF2 (SC-136999), -TRAF6 (SC-8409), tissue plasminogen activator (tPA) inhibitor were from Santa Cruz Biotechnology, Inc. (Santa Cruz, CA). Seize-X immunoprecipitation kit, antigen elution buffer, BindTM NeutrAvidinTM, high binding capacity coated 96-well plates, West pico chemiluminescent reagents, Superblock blocking agents and Fermentas PageRuler Pre-stained Protein Ladder were purchased from Thermo Pierce (Rockford, IL). Bradford reagent, SDS-PAGE reagents, and Precasted IEF pH3-10 gels were from Bio-Rad Laboratories (Hercules, CA). Protease inhibitors (EDTA-free) and protein phosphatase inhibitor (PhosSTOP) tablets were purchased from Roche (Mannheim, Germany). MMP-9 inhibitor I was purchased from EMD Biosciences/Calbiochem (San Diego, CA).

BDNF was reconstituted to 10 ng/μl concentrations by following the manufacturer’s instructions with 10% glycerol added to minimize freezing damages and stored in -80°C until use. All other test agents were made fresh according to the manufacturer’s recommendation. The content of DMSO in the incubation medium was ≤ 1%.

### Animal treatment

All animal treatment and experimental procedures were strictly adhered to the National Institutes of Health Guide for Care and Use of Laboratory Animals and were approved by the City College of New York Animal Care and Use Committee. Pregnant female Sprague-Dawley rats weighing about 200-215g were purchased from Taconic (Germantown, NY). Following acclimatization, the rats were individually housed in a 12 h light/dark cycle with *ad libitum* access to food and water but without disturbance to the animals other than a daily injection of cocaine or saline. From gestation days 8–21, pregnant dams received daily intraperitoneal injections of either 30 mg/kg cocaine HCl in 0.9% saline (30 mg cocaine HCl/ml) or 2 ml/kg saline between 10–11 a.m. To minimize skin lesions in the cocaine-injected rats, the injection sites were alternated every other day. To reduce the risk of increased extraplacental absorption of cocaine, intraperitoneal injections were administered with tuberculin syringe and away from the womb. Following each injection, pregnant rats were observed for 1 h and behavioral abnormalities were recorded. There were apparent increases in locomotor activity in cocaine-treated rats. However, there were no discernible differences in litter size (7–13 pups), in body weight of the pups at 21 days of age prior to sacrifice (45.9 ± 2.6 and 51.8 ± 2.7 g for cocaine and saline, respectively; *n* = 40 each), or in gender distribution (23 males/17 females and 19 males/21 females for cocaine and saline groups, respectively). There were no apparent changes in rearing behaviors and more importantly, the dose of cocaine used did not cause seizure or fatality throughout the treatments.

RETRACTED

Progeny were cross-fostered and group housed with treatment-naïve surrogate mothers until they were sacrificed at 21 days of age (P21). Because neurotrophins play an important role in regulating dendritic dynamics and excitatory neurotransmission, and because we observed significant changes in dendritic spin morphology [7] and AMPAR transmission/signaling [21] in our previous rodent studies using P21 rats (an age when adult excitatory glutamatergic receptors are found), we selected P21 so that this investigation can also assess crosstalk between neurotrophin and NMDAR systems. Food and water were freely available. Rats were subjected to the minimum handling associated with routine animal husbandry. Since we did not find gender differences in our earlier studies conducted in rabbit and rats [7],[8],[21], both sexes from separate litters were employed in these experiments. To prevent oversampling, only one pup from each litter was used in each experiment [22].

### Brain slices preparation

Rats were sacrificed by rapid decapitation and brains were dissected on ice. The olfactory bulbs were removed, a coronal cut was made at +4 mm rostral of the optical chiasm and the anterior portion was taken as the prefrontal cortices (PFCX). The caudal portions of the cortices were gently peeled laterally from the midline to expose the hippocampi.

Slices were prepared as described in our earlier report [23]. Briefly, brain slices were cut using a chilled McIlwain tissue chopper into 100 μm x 100 μm x 3 mm slices. Approximately 10 mg of brain slices were suspended in 1 ml of ice-cold oxygenated low Mg^2+^ Kreb’s-Ringer (LMKR), containing 25 mM HEPES, pH7.4, 118 mM NaCl, 4.8 mM KCl, 1.3 mM CaCl_2_, 1.2 mM KH_2_PO_4_, 0.3 mM MgSO_4_, 25 mM NaHCO_3_, 10 mM glucose, 100 μM ascorbic acid, 50 μg/ml leupeptin, 0.2 mM PMSF, 25 μg/ml pepstatin A, and 0.01 U/ml soybean trypsin inhibitor. Brain slices were collected following brief centrifugation at 4°C and were washed twice more and then suspended in 1 ml oxygenated LMKR.

RETRACTED

### Preparation of synaptosomes

Synaptosomes (P2 fraction) were prepared from frontal cortices as previously described with few modifications [23]. To further purify synaptosomal factions, the synaptosome-enriched P2 fraction was washed twice in 5 ml of oxygenated ice-cold Kreb’s-Ringer solution (K-R): 25 mM HEPES, pH 7.4; 118 mM NaCl, 4.8 mM KCl, 25 mM NaHCO_3_, 1.3 mM CaCl_2_, 1.2 mM MgSO_4_, 1.2 mM KH_2_PO_4_, 10 mM glucose, 100 μM ascorbic acid, 50 μg/ml leupeptin, 10 μg/ml aprotinin, 2 μg/ml soybean trypsin inhibitor, 0.04 mM phenylmethylsulfonyl fluoride (PMSF), 0.1 mM 2-mercaptoethanol, 10 mM NaF, 1 mM Na_3_VO_4_ and protein phosphatase inhibitors. To obtain cytosolic and membranous fractions of the synaptosomes, the washed synaptosomes were sonicated for 10 s on ice in 0.5 ml hypo-tonic homogenization solution (25 mM HEPES, pH 7.4; 12 mM NaCl, 0.5 mM KCl, 2.5 mM NaHCO_3_, 0.1 mM CaCl_2_, 0.1 mM MgSO_4_, 0.1 mM KH_2_PO_4_, 1 mM glucose, 10 μM ascorbic acid, 50 μg/ml leupeptin, 10 μg/ml aprotinin, 2 μg/ml soybean trypsin inhibitor, 0.04 mM PMSF and 0.1 mM 2-mercaptoethanol, 10 mM NaF, 1 mM Na_2_VO_4_ supplemented with protein phosphatase inhibitor cocktail (PhosSTOP tablet, Roche). Samples were then centrifuged at 50,000 x g for 30 min. The resultant supernatant was taken as the cytosolic fraction and the synaptic membrane pellet resuspended in 0.5 ml of LMKR. Protein concentrations of the synaptic membranes were determined using the Bradford method (Bio-Rad) and used as the tissue source for determination of levels of BDNF-induced TrkB and p75^NTR^ signaling.

### Assessments of *ex vivo* tissue treatment on BDNF-TrkB signaling and TrkB-NMDAR association

To assess the effects of prenatal cocaine exposure on TrkB signaling in brain tissues, brain slices were incubated for 30 min at 37°C in 0.5 ml oxygenized LMKR with or without 50 ng/ml rhBDNF (for BDNF—TrkB signaling). A preliminary experimental series that measured the dose-response relationship of BDNF to the activation of TrkB found the ED50 for stimulating TrkB to be 50 ng/ml of BDNF. To confirm that 50 ng/ml rhBDNF activates TrkB signaling preferentially, TrkB and p75^NTR^ signaling were determined in tissues incubated with 50, 100 and 200 ng/ml of rhBDNF.

Using a method similar to that of our earlier study [23], the reaction mixture was oxygenated with 95% O_2_/5% CO_2_ for 1 min every 10 min during incubation. Ligand stimulation was stopped by adding 1 ml of ice-cold Ca^2+^-free LMKR containing 0.5 mM EGTA/0.1 mM EDTA and phosphatase inhibitors, and centrifuged briefly. Supernatant was discarded and tissue slices were homogenized in 0.25 ml ice-cold immunoprecipitation buffer (25 mM HEPES, pH 7.5, 200 mM NaCl, 1 mM EDTA, 50 μg/ml leupeptin, 10 μg/ml aprotinin, 2 μg/ml soybean trypsin inhibitor, 0.04 mM PMSF, 5 mM NaF, 1 mM sodium vanadate, 0.5 mM β-glycerophosphate, and 0.02% 2-mercaptoethanol containing 0.5% digitonin, 0.2% sodium cholate, and 0.5% NP-40. The resulting homogenates were centrifuged at 1000g for 5 min (4°C), the supernatant (post-mitochondrial fraction) sonicated for 10 s on ice, and protein concentrations measured by the Bradford method (Bio-Rad). We solubilized 200 μg of lysate in 0.5% digitonin/0.2% sodium cholate/0.5% NP-40 for 60 min at 4°C via end-to-end rotation. Resultant lysates were cleared by centrifugation at 50,000g for 5 min and suspended in 100 μl of immunoprecipitation buffer.

RETRACTED

### Determination of TrkB activation by the recruitment of phospholipase C-γ1, shc, and N-shc to TrkB; TrkB-NMDAR interaction; p75^NTR^ association with TRAF2 and TRAF6; and ERK and PI3K activation using co-immunoprecipitation technique

Using the method described in our earlier work [23], TrkB signaling complexes, ERK2 and Akt were immunopurified separately from 200 μg of tissue lysate. Briefly, 200 μg of tissue lysate was incubated at 4°C for 2 h with 1 μg immobilized anti-TrkB (for assessment of pY-TrkB; phospholipase C-γ1 (PLC-γ1), shc and N-shc recruitment; and TrkB–NMDAR interaction); 1 μg immobilized anti-ERK2 (pT^202^/ pY^204^-ERK2), or 1 μg immobilized mouse anti-Akt1 (pS^473^-Akt) followed by addition of 30 μl protein A/G-conjugated agarose beads. Incubation continued at 4°C for 16 hr. The immunocomplexes were centrifuged at 4°C and the immunoprecipitates were washed three times with 1 ml 0.05% NP-40 containing ice-cold PBS (pH 7.2) and centrifuged. The resultant immunoprecipitates were solubilized by boiling in 100μl SDS-PAGE sample preparation buffer (62.5 mM Tris-HCl, pH 6.8, 10% glycerol, 2% SDS, 5% 2-mercaptoethanol, and 0.1% bromophenol blue) for 5 min. The levels of pY-TrkB, PLC-γ1, shc, N-shc, and NMDAR subunits in 50% of anti-TrkB immunoprecipitate, pT^202^/ pY^204^-ERK2 in 50% anti-ERK2 immunoprecipitate, and pS^473^Akt1 in 50% anti-Akt1 immunocomplexes were assessed by Western blotting. The blots were stripped and re-probed with anti-TrkB, -ERK2, or -Akt1/2/3 to demonstrate even immunoprecipitation efficiency and loading.

P75^NTR^ signaling was assessed by its interaction with TRAF2 and TRAF6 [24]. Briefly, p75^NTR^ and its associated proteins TRAF2 and TRAF6 were immunoprecipitated in 200 μg of tissue lysate for a 2-h incubation (4°C) with 1 μg of immobilized anti-p75^NTR^ followed by addition of 30 μl protein A/G-conjugated agarose beads. Incubation continued at 4°C for 16 hr. The resultant immunocomplexes were pelleted by centrifugation (4°C), washed three times with 1 ml ice-cold PBS (pH 7.2) and centrifuged. The resultant immunocomplexes were solubilized by boiling for 5 min in 100μl of SDS-PAGE sample preparation buffer and the contents of the TRAF2 and TRAF6 in 50% anti-p75^NTR^ immunoprecipitate were determined by Western blotting. The blots were stripped and re-probed with anti-p75^NTR^ to ascertain similar immunoprecipitation efficiency and loading.

RETRACTED

### Western blot analysis

The Western blotting procedure was performed using the method described earlier [23]. Briefly, solubilized immunoprecipitates, size-fractionated by either 7.5 or 10% SDS-PAGE, were electrophoretically transferred to nitrocellulose membranes. The membranes were washed with PBS and blocked overnight at 4°C with 10% milk in 0.1% Tween 20-containing PBS (PBST). Following three 5-min washes with 0.1% PBST, membranes were incubated at 25°C for 2 h with 1:500 to 1:1,000 dilutions of selected antibodies. After three 2-min 0.1% PBST washes, membranes were incubated for 1 h with anti-species IgG-HRP (1:5000 dilution) and washed three times with 0.1% PBST for 2 min each. The signals were detected using a chemiluminescent method and visualized by exposure to x-ray film. Specific bands were quantified by densitometric scanning (GS-800 calibrated densitometer, Bio-Rad).

### BDNF binding

We used synaptosomes prepared from hippocampi and PFCX of prenatal cocaine- and saline-exposed P21 rats to assess BDNF binding. Membrane-bound proteins in the synaptosomes were first biotinylated using a biotinylation kit. The biotinylated surface proteins containing synaptosomes were sonicated in 500 μl LMKR for 10 s on ice and solubilized by 0.5% digitonin/0.2% sodium cholate/0.5% NP-40 and diluted 1:5. Protein concentrations were measured using the Bradford method. The biotinylated protein solution was diluted with LMKR to 50 μg/100 μl. To coat the plate with biotinylated proteins, streptavidin-coated plates (Reacti-Bind NeutrAvidin high binding capacity 96-well plates) were washed three times with 200 μl of ice-cold LMKR and incubated at 30°C with 50 μg/well biotinylated receptor solution for 1 h in the presence of 5% blocking reagent. Following two LMKR washes, BDNF was added (100 fM to 10 nM), and incubation was performed at 30°C for 1 h. Plates were washed with ice-cold LMKR and incubated at 30°C for 1 h with anti-BDNF (0.5 μg/well) in PBST, followed by FITC-conjugated anti-rabbit IgG (0.05 μg/well) in PBST for 1 h. Plates were washed twice with 200 μl of ice-cold PBST and then twice with 200 μl PBS, and the FITC signals were determined by a multimode plate reader, DTX880 (Beckman). Negligible FITC signal was noted when vehicle was added. Nonlinear regression data curve fit was performed using Prism.

RETRACTED

### Isoelectric point assessment

To purify TrkB, hippocampus and PFCX synaptosomes of prenatal saline- or cocaine-exposed P21 rats were sonicated for 10 s on ice and solubilized using 0.5% digitonin/0.2% sodium cholate/0.5% NP-40 at 4°C with end-over-end rotation for 1 hr. Following centrifugation to remove insoluble debris, the obtained lysate was treated with 1% SDS for 1 min to dissociate the TrkB-associated proteins, diluted 10-fold with immunoprecipitation buffer, and imunopurified with immobilized anti-TrkB. The resultant TrkB (145- and 95-KDa) was eluted using 200 μl antigen-elution buffer (Thermo), neutralized immediately with 100 mM Tris HCl (pH9.0), diluted to 500 μl with 50 mM Tris HCl, pH7.5, and passed through a 100 kD cut-off filter to remove 95-KDa TrkB isoform. Once purified, the 145-KDa TrkB was suspended in 100 μl isoelectric focusing sample buffer. Samples (50 μl) were loaded onto pH 3–10 isoelectric focusing gels and the proteins were fractionated (100 V for 1 hr, 200 V for 1 hr, and 500 V for 30 min). The separated proteins were then electrophoretically transferred to nitrocellulose membranes. TrkB was identified by Western blotting with anti-TrkB.

### BDNF and proBDNF release

BDNF and proBDNF release was determined in hippocampal and PFCX slices (100 μl x 100 μl x 3 mm) from prenatal cocaine- and saline-exposed P21 rats. Brain slices of approximately 10 mg were suspended in 250 μl oxygenized LMKR and loaded onto a superfusion chamber and superfused at 0.2 ml/min with oxygenated LMKR at 37°C for 30 min. Spontaneous (basal) BDNF/proBDNF efflux was defined by the levels of BDNF/proBDNF in LMKR perfusate at the 30-min mark. Depolarization- and NMDA (10 μM)/glycine(1 μM)-induced (stimulated) BDNF/proBDNF release was evoked by superfusion of brain slices with 65 mM K^+^ (NaCl replaced with KCl) for 1 min followed by LMKR or LMKR-containing NMDA(10 μM)/glycine (1 μM) for 9 min. Next, brain slices were superfused with oxygenated LMKR at 37°C for 20 min and collected at the conclusion of superfusion. For the proBDNF release with minimal proteolytic conversion to BDNF, brain slices were treated with 10 μM of MMP-9 inhibitor I and tissue plasminogen activator (tPA) inhibitor for 10 min and superfused with 0.2 ml/min LMKR containing 10 μM MMP-9 and tPA inhibitors as described above.

To assess levels of BDNF and proBDNF in the perfusate (6 ml), protease inhibitors and detergents (digitonin/sodium cholate/NP-40) were first added to the perfusate to achieve final concentrations of 0.05% digitonin/0.02% sodium cholate/0.05% NP-40). BDNF and proBDNF were immunoprecipitated with anti-BDNF (1 μg/ml) followed by protein A/G-conjugated agarose beads. The levels of BDNF and proBDNF were measured using Western blotting with anti-BDNF and anti-proBDNF. To assess the percentage of brain tissue from which BDNF/proBDNF was released, tissue slices were homogenized and diluted 10-fold in immunoprecipitation buffer. Following centrifugation at 1000g for 10 min, the resultant supernatant (post-mitochondrial fraction) was used to measure protein content by the Bradford method and solubilized by boiling in sample preparation buffer for 5 min. The level of β-actin was measured by Western blotting to control for tissue quantity.

RETRACTED

### Statistical analyses

All data are presented as mean ± s.e.m. and the treatment effects were evaluated first by ANOVA, as in our earlier study [23]. Treatment effects on TrkB activation-related biochemical indices in the current investigation were evaluated by Newman-Keul’s test for multiple comparisons or by two-tailed Student’s t test, as appropriate. The threshold for significance was p < 0.05. Between-group comparisons were also conducted for all parameters.

## Results

### Prenatal cocaine exposure enhances BDNF-TrkB signaling without affecting basal expression of BDNF, TrkB, P75^NTR^ and downstream signaling components for TrkB

Total expression of BDNF, proBDNF, full length TrkB (145-KDa) and truncated TrkB (95-KDa), p75^NTR^, NMDAR-NR1 as well as the constituents of the TrkB signaling cascade including N-Shc and shc, Akt1 and ERK2 were determined by Western blotting in the tissue lysates of PFCX and hippocampi from 2 male and 2 female prenatal saline-treated (n = 4) and cocaine-exposed (n = 4) P21 rats (Fig 1). *In utero* cocaine exposure did not affect the levels of 145-KDa (full-length) and 95-KDa (truncated) forms of TrkB (a), p75^NTR^ (b), BDNF and proBDNF (c). Similarly, prenatal cocaine exposure did not influence the expression levels of the TrkB signaling components including Akt1 and ERK2 (d), Shc and N-Shc (e) as well as phospholipase C-γ1 (f) and NMDAR-NR1 subunit. There was also no discernible gender difference in the levels of all the proteins tested.

**Fig 1:** Prenatal cocaine exposure did not alter the expression levels of full-length (145-KDa) and truncated (95-KDa) TrkB, p75^NTR^, pro-BDNF and BDNF, Akt1 and ERK2, N-Shc and Shc, as well as NR1 and PLC-γ1 in both hippocampus and prefrontal cortex. The expression levels of 145- and 95-KDa TrkB (a). P75NTR (b), pro-BDNF and BDNF (c) as well as Akt1 and ERK2(d), Shc and N-Shc (e), NR1 and PLC-γ1(f), in 50 μg post-mitochondrial synaptosome-enriched fractions prepared from hippocampi and PFCX of P21 rats exposed to saline or cocaine *in utero* were compared by Western blotting. The blots were stripped and re-probed with anti-β-actin to validate equal loading. Densitometric quantification of blots revealed no discernible differences in 145- and 95-KDa TrkB, P75NTR, proBDNF and BDNF, Akt1, ERK2, Shc and N-Shc, NR1 and PLC-γ1 expression levels. n = 4. Data are mean ± s.e.m. of the ratio of 145-, 95-KDa TrkB, p75^NTR^, proBDNF, BDNF, Akt1, ERK2, N-Shc, Shc, NR1 or PLC-γ1to β-actins optical intensities.

RETRACTED

Because there is an extensive functional interaction between TrkB and p75^NTR^, we first examined the effect of *ex vivo* exposure to varying concentrations of BDNF on the expression of 145-KDa and 95-KDa TrkB as well as p75^NTR^. Incubation of either hippocampal or PFCX slices from 2 male and 2 female prenatal saline-treated (n = 4) and cocaine-exposed (n = 4) P21 rats with 50–200 ng/ml of BDNF for 30 min had no discernible effects on expression levels of the 145-KDa or 95-KDa TrkB or p75^NTR^ (Fig 2). Exposure to BDNF also did not affect the cellular distribution of the 145-KDa and 95-KDa TrkB: over 90% of the full-length and truncated TrkB as well as p75^NTR^ were found in the membranes of the synaptosomes prepared from PFCX and hippocampi of both prenatal cocaine- and saline-exposed rats (data not shown).

**Fig 2:** *Ex vivo* exposure to 50–200 ng/ml BDNF did not alter the expression of full-length (145-KDa) and truncated (95-KDa) TrkB and p75NTR in BDNF-incubated hippocampal and prefrontal cortical slices. The abundance of 145- and 95-KDa TrkB (a, b) as well as p75NTR (c, d) in 50 μg post-mitochondrial synaptosome-enriched fractions prepared from hippocampal and PFCX slices of P21 prenatal cocaine- and saline-exposed rats following 30-min incubation with 50–200 ng/ml BDNF were compared by Western blotting. The blots were stripped and re-probed with anti-β-actin to validate equal loading. Densitometric quantification of blots revealed no discernible differences in 145- and 95-KDa TrkB as well as p75NTR expression levels as a result of incubation with BDNF. n = 4. Data are mean ± s.e.m. of the ratio of 145-, 95-KDa TrkB, p75NTR to β-actin optical intensities.

Next we examined whether TrkB and p75^NTR^ are differentially activated under current experimental conditions. The data summarized in Fig 3 show that although 50–200 ng/ml BDNF activates 145-KDa TrkB dose-dependently, as indicated by the elevated pY-145-KDa TrkB levels [Hippocampus: *F*(3, 12) = 104.93, p < 0.00001; PFCX: F(3,12) = 115.99, p < 0.00001], BDNF was not only less effective in activating 95-KDa TrkB but also dose-insensitive in both hippocampi and PFCX [Hippocampus: *F*(3, 12) = 67.16, p < 0.00001; PFCX: F(3,12) = 95.45, p < 0.00001] (Fig 3). By contrast, p75^NTR^ activation, indicated by the recruitment of TNF receptor-associated factor 2 (TRAF2) and TNF receptor-associated factor 6 (TRAF6) to p75^NTR^, was observed only at 200 ng/ml BDNF [Hippocampus: TRAF6: *F*(3, 12) = 139.70, p < 0.00001, at 200 ng/ml BDNF: t(4) = 7.3482, p = 0.00183, TRAF2:; PFCX: *F*(3,12) = 63.32, p < 0.00001, at 200 ng/ml BDNF: t(4) = 10.4010, p = 0.00048; PFCX: TRAF6: *F*(3, 12) = 49.23, p < 0.00001, at 200 ng/ml BDNF: t(4) = 7.8078, p = 0.00145, TRAF2: *F*(3,12) = 55.74, p < 0.00001, at 200 ng/ml BDNF: t(3) = 9.3508, p = 0.00259] (Fig 3). These data indicate that BDNF-TrkB signaling induced by the 50 ng/ml BDNF *ex vivo* exposure is not the result of increased TrkB expression and is relatively free of interference from p75^NTR^ activation.

RETRACTED

**Fig 3:** The concentration-response relationships of BDNF-induced TrkB and p75^NTR^ activation. Concentration-response relationships of BDNF-induced TrkB and p75^NTR^ activation indicate that p75^NTR^ is far less sensitive to BDNF than TrkB. (a) The magnitudes of TrkB and p75NTR activation induced by a 30-min incubation with 50–200 ng/ml BDNF were assessed in hippocampal and PFCX slices prepared from naïve P21 rats using pY TrkB and TRAF2/6 recruitment to p75^NTR^, respectively, as the guides. (b) Densitometric quantification of pY 145- and 95-KDa TrkB and TRAF2/6 blots revealed that while TrkB was activated by 50–200 ng/ml of BDNF in a dose-dependent manner, p75NTR is activated only by 200 ng/ml of BDNF in both hippocampus and PFCX. n = 4. Data are mean ± s.e.m. of the ratios of pY to total 145-, 95-KDa TrkB or TRAF2 and TRAF6 to p75^NTR^ optical intensities. *p < 0.01 compared to the basal level of respective protein.

Incubation of PFCX and hippocampal slices with exogenous 50 ng/ml of human BDNF resulted in 4.5-7-fold and 4-fold increases in levels of activated (tyrosine-phosphorylated, pY) 145- and pY 95-KDa TrkB, respectively, in both hippocampus and PFCX of saline-exposed rats. In the prenatal cocaine exposed group, BDNF-induced pY-145-KDa TrkB was 222% [t(7) = 8.5167, p < 0.00001] and 196% [t(7) = 5.7451, p = 0.00019] of that of the saline-exposed group in the hippocampus and PFCX, respectively (Fig 4). In contrast, levels of BDNF-induced pY-95-KDa dominant-negative, truncated TrkB were similar in hippocampi [t(9) = 1.1624, p = 0.27498] or slightly increased in prefrontal cortices [t(9) = 3.3988, p = 0.00363] of the prenatal cocaine- compared to saline-exposed P21 rats (Fig 4).

RETRACTED

**Fig 4:** Prenatal cocaine exposure increased 50 ng/ml BDNF-induced TrkB activation in hippocampi and PFCX. (a) Representative blots showing prenatal cocaine exposure increased 50 ng/ml BDNF-induced TrkB activation in hippocampi and PFCX evidenced by higher activated (tyrosine-phosphorylated [pY]) TrkB. (b) Summary of the densitometric quantification of the pY and total 145- and 95-KDa TrkB. The data are expressed as the ratios of pY- full-length (145-KDa) and truncated TrkB (95-KDa) optical intensity normalized by the optical intensity of total 145- and 95-KDaTrkB, respectively. n = 6 (3 females and 3 males). Data are reported as means ± s.e.m. of the ratio of pY-TrkB to TrkB optical intensities. *p < 0.01, **p < 0.05 compared to respective protein in the saline-treated group.

The finding of a higher BDNF-induced pY-145-KDa TrkB in prenatal cocaine exposed brains was substantiated by higher levels of BDNF-induced recruitment of phospholipase C-γ1 (173% [t(6) = 5.0262, p = 0.00262] and 86% [t(6) = 7.6590, p < 0.00001] increase in hippocampus and PFCX, respectively) and adaptor proteins Shc (70% [t(8) = 7.5245, p < 0.00001] and 50% [t(8) = 6.0854, p = 0.00029] increase in hippocampus and PFCX, respectively) and N-Shc (91% [t(9) = 4.9070, p = 0.00089] and 42% [t(10) = 4.0074, p = 0.00249] increase in hippocampus and PFCX, respectively) to specific pY-TrkB docking sites (Fig 5a). Additional evidence of enhanced 145-KDa TrkB activation was corroborated by the increased activation of its downstream signaling pathways. BDNF-induced PI3K and ERK2 activation was indicated by increases in pS^473^Akt1 (55% [t(10) = 10.0014, p < 0.00001] and 73% [t(8) = 4.9124, p < 0.00118] in hippocampus and PFCX, respectively; Fig 5b) and in pT^202^/pY^204^-ERK2 (59% [t(8) = 7.3778, P < 0.00001] and 59% [t]7) = 6.8395, P = 0.00025] in hippocampus and PFCX, respectively; Fig 5c) in prenatal cocaine-exposed brains.

**Fig 5:** Prenatal cocaine increases BDNF-induced phospholipase C-γ1, Shc and N-Shc recruitment to the activated TrkB as well as downstream PI3K and ERK2 activation in hippocampus and PFCX. (**a**) Prenatal cocaine exposure increased 50 ng/ml BDNF-induced recruitment of the downstream signaling molecules phospholipase C-γ1, and adaptor proteins, Shc and N-Shc to activated TrkB in hippocampus and PFCX. Western blots of phospholipase C-γ1, N-Shc, and Shc as well as TrkB that served as the loading control were analyzed by densitometric quantification. Data are means ± s.e.m. of the ratios of phospholipase C-γ1, N-Shc, or Shc to TrkB optical intensities. n = 6 (3 males and 3 females). Prenatal cocaine exposure also enhanced PI3K and ERK signaling downstream of TrkB in hippocampus and PFCX as evidenced by the Western blot detection of increased activated (pS^473^)- Akt1 (**b, top**) and (pT^202^/pY^204^)-ERK2 (**c, top**). Densitometric quantification of blots is shown in the bottom of the representative blot. Data are means ± s.e.m. of the ratios of pS^473^-Akt1/Akt1 (**b, bottom**) and pT^202^/pY^204^-ERK2/ERK2 (**c, bottom**) optical intensities. n = 6 (3 males and 3 females). *p < 0.01, compared to respective protein in the saline-treated group.

RETRACTED

BDNF-TrkB activation can regulate long-term synaptic plasticity by interacting with NMDARs. To assess whether gestational cocaine exposure affects the inter-relationship between activated TrkB and NMDARs, we measured the levels of the obligatory NMDAR subunit, NR1, that co-immunoprecipitated with TrkB with or without BDNF incubation. Our results show that BDNF stimulation increased the level of TrkB-NMDAR association in brain regions from both prenatal cocaine- and saline-exposed P21 rats as indicated by a marked increase in NR1 in anti-TrkB immunoprecipitates. While there was no discernible difference in TrkB-NMDAR complex level under basal conditions, prenatal cocaine exposure increased BDNF-induced TrkB association with NMDARs by 56% [t(6) = 5.3325, p = 0.00033] in the hippocampus and by 49% [t(7) = 5.0283, p = 0.00015] in PFCX above that of the saline-treated group (Fig 6).

**Fig 6:** Prenatal cocaine exposure heightened TrkB-NMDAR interaction in hippocampi and PFCX. Prenatal cocaine exposure heightened TrkB-NMDAR interaction in hippocampi and PFCX as indicated by the Western blot detection of increased level of obligatory subunit of the NMDARs, NR1 in the anti-TrkB immunoprecipitates (top). Western blots were analyzed by densitometric quantification. The data are expressed as the ratios of NR1 optical intensity normalized by the optical intensity of total 145-KDa TrkB. n = 6 (3 males and 3 females). Data are means ± s.e.m. of the ratios of NR1 to 145-KDa TrkB optical intensities. *p < 0.01, compared to respective protein in the saline-treated group.

Collectively, these data indicate that prenatal cocaine exposure heightens the efficacy of BDNF-TrkB signaling and improves the interaction between activated TrkB and NMDAR complexes.

### Enhanced BDNF binding affinity for TrkB is responsible for prenatal cocaine-induced increases in BDNF-TrkB signaling

Next, we attempted to resolve the underlying mechanism responsible for the heightened BDNF-TrkB signaling (Figs 3–5) and heightened BDNF-TrkB/NMDARs interaction (Fig 6). Because prenatal cocaine exposure did not affect TrkB expression level, we tested whether prenatal cocaine exposure affects the affinity of BDNF for TrkB. Similar to the method described earlier [23], biotinylated surface receptors were used as the tissue source for the BDNF binding assessments by a modified binding assay with fluorescence detection. Our results show that the BDNF saturation curves in brain areas from both prenatal cocaine- and saline-exposed P21 rats fit significantly better when the nonlinear regression curve-fit algorithm assumed the presence of two saturation sites rather than one, presumably reflecting the presence of TrkB and p75NTR (r 2 > 0.911). The calculated Kd values for the prenatal saline-exposed brains were 11.8 pM and 60.8 nM in hippocampus and 3.9 pM and 21.9 nM in PFCX. Prenatal cocaine exposure increased BDNF binding affinities at the high-affinity binding sites by 17.8- and 15-fold in hippocampus and PFCX, respectively, to 0.66 pM and 0.26 pM. Moreover, prenatal cocaine exposure improved BDNF affinities at the low-affinity binding sites by 80.1- and 12-fold in hippocampus and PFCX, respectively, to 0.74 nM and 1.86 nM (Fig 7). These data strongly suggest that an increased BDNF binding affinity is responsible for more efficacious BDNF-TrkB signaling in prenatal cocaine-exposed brains.

RETRACTED

**Fig 7:** Prenatal cocaine exposure increased BDNF binding affinity for TrkB. Prenatal cocaine exposure increased BDNF binding affinity for TrkB by 18- and 15- fold (dotted lines) in biotinylated hippocampal and PFCX synaptic membranes, respectively from P21 prenatal cocaine- and saline-treated rats. In the control membranes, there were two BDNF binding sites, a high-affinity site (KD1) and a low-affinity site (KD2) (solid lines). Prenatal cocaine exposure also increased the low-affinity binding of BDNF by 82- and 12-fold. Nonlinear regression data curve fit was performed using Prism. Data points are the means and vertical bars are the s.e.m. derived from 6 independent rats (3 males and 3 females) in each treatment group.

### Prenatal cocaine-exposure elicits a conformational change in TrkB as reflected by a shift in isoelectric point

To determine whether conformational changes in TrkB in the prenatal cocaine-exposed brains contribute to enhanced BDNF binding affinity for TrkB, we individually isolated TrkB by immunoprecipitation using immobilized anti-TrkB from the hippocampus and PFCX lysates. Following elution, the TrkB-containing eluate was passed through a 100-KDa molecular weight cut-off filter to remove the 95-KDa truncated TrkB. The isoelectric point (pI) of TrkB was determined by separation on isoelectric-focusing gels followed by Western blotting. The results summarized in (Fig 8) indicate that prenatal cocaine exposure causes a shift in TrkB’s calculated pI from 6.1 to 6.9 in both hippocampus [t(6) = 20.9835, p < 0.00001] and PFCX [t(6) = 35.9368, p < 0.00001]. The data therefore suggest that conformational changes in TrkB contribute to the observed increases in affinity of BDNF for TrkB.

RETRACTED

**Fig 8:** Prenatal cocaine exposure altered 145-KDa TrkB conformation in hippocampi (top) and PFCX (bottom). The conformational states of the immunopurified 145-KDa TrkB was analyzed by separating on pH3-10 isoelectric focusing gels and then Western blotted with anti-TrkB. Blots were quantified by densitometric scanning. Data are means ± s.e.m. of the pI 6.1 and pI 6.9. n = 5 (3 males and 2 females). p < 0.01 compared to respective protein in the saline-treated group.

### Prenatal cocaine decreases endogenous proBDNF and BDNF release

BDNF-TrkB signaling is an important regulator of long-term plasticity and function of the glutamatergic synapses. In turn, BDNF release is triggered and regulated by glutamatergic synaptic activity. BDNF can be released from both presynaptic terminals and postsynaptic dendritic fields [23, 25–26]. To further probe the underlying mechanism responsible for the upregulated BDNF-TrkB signaling and the BDNF affinity for TrkB, we explored the potential contribution of altered BDNF/proBDNF release from both presynaptic terminals and postsynaptic dendritic fields using K^+^-depolarization and NMDA/glycine. Endogenous BDNF release was evoked by 65 mM K^+^-depolarization, presumably from the presynaptic axonal terminals or by 10 μM NMDA/1 μM glycine, presumably from the postsynaptic dendritic field in both hippocampus and PFCX (Fig 9). Prenatal cocaine exposure did not have a discernible effect on spontaneous BDNF and proBDNF efflux in either brain region. In response to K^+^-depolarization and NMDA/glycine, BDNF and proBDNF in the perfusate increased markedly by approximately 6- and 4-fold, respectively, in the hippocampus and PFCX of the prenatal saline-exposed control rats. The stimulated BDNF and proBDNF release was reduced in prenatal cocaine-exposed P21 rats by 50–60% in the hippocampi [fold increases in BDNF: t(4) = -3.3142, p = 0.04525 by K^+^, t(4) = -5.7900, p = 0.01025 by NMDA/glycine; fold increases in proBDNF: t(4) = -3.1394, p = 0.02568 by K^+^, t(4) = -3.4097, p = 0.02703 by NMDA/glycine] and PFCX fold increases in BDNF: t(4) = -3.5962, p = 0.02284 by K^+^, t(4) = -6.1707, p = 0.00350 by NMDA/glycine; fold increases in proBDNF: t(4) = -3.4258, p = 0.01404 by K^+^, t(4) = -2.7508, p = 0.04027 by NMDA/glycine] (Fig 9). The levels of the 32-kDa proBDNF were markedly lower than the 14-kDa mBDNF form, indicating that most of the proBDNF was converted to mBDNF within the timeframe of the test.

RETRACTED

**Fig 9:** Prenatal cocaine exposure reduced NMDA/Glycine and K^+^-depolarization induced BDNF and proBDNF release in hippocampi (a) and PFCX (b). Hippocampal and PFCX slices prepared from P21 prenatal cocaine- and saline-treated rats were used to determine spontaneous BDNF/proBDNF efflux as well as BDNF and proBDNF release induced by 10-min 10 μM NMDA/1 μM glycine in LMKR or 1-min 65 mM K^+^-depolarization in a superfusion system. BDNF and proBDNF in the perfusate were then immunoprecipitated with immobilized anti- BDNF and determined by Western blotting with anti-BDNF. The brain slices were collected, homogenized and solubilized and the level of β-actin in the brain slices was determined by Western blotting to illustrate equal quantities of tissues. The blots were quantified by densitometric scanning. Data are expressed as means ± s.e.m. of the ratios of BDNF or proBDNF optical intensity to the optical intensity of β-actin. n = 6. **p < 0.05, *p < 0.01 compared to LMKR-treated in the same group. ##p < 0.05, #p < 0.01 compared to respective protein in the saline-treated group.

Since MMP-9 and tPA are the primary proteases that convert proBDNF to mBDNF, we investigated whether the effect of prenatal cocaine exposure on the release of mBDNF is the result of reduced activity of these factors. To this end, brain slices were incubated with and superfused in the presence of metalloprotease (MMP-9) and tissue plasminogen activator (tPA) inhibitors prior to the induction of proBDNF release by K^+^-depolarization or 10 μM NMDA + 1 μM glycine. K^+^-depolarization and NMDA/glycine markedly increased proBDNF in the perfusate by approximately 3.5–5.5 folds in the hippocampus and PFCX of prenatal saline-exposed P21 control rats with minimal mBDNF detected (data not shown). Prenatal cocaine exposure decreased proBDNF release by these stimuli by 51–55% in hippocampi [fold increases: t(4) = -3.0614, p = 0.03761 by K^+^, t(4) = -4.2108, p = 0.00840 by NMDA/glycine] and PFCX [fold increases: t(4) = -2.9737, p = 0.04100 by K^+^, t(4) = -7.5242, p = 0.00066 by NMDA/glycine] (Fig 10).

**Fig 10:** Prenatal cocaine exposure reduced proBDNF release in hippocampi (top) and PFCX (bottom). Brain slices treated with 10 μM of MMP-9 inhibitor I and tPA inhibitor were used to assess proBDNF released spontaneously and induced by 10-min 10 μM NMDA/1 μM glycine or 1-min 65 mM K^+^-depolarization. ProBDNF in the perfusate were then immunoprecipitated with immobilized anti-BDNF and the level of proBDNF was determined by Western blotting with specific anti-proBDNF. The brain slices were collected, homogenized, and solubilized and the level of β-actin in the brain slices was determined by Western blotting. The blots were quantified by densitometric scanning. Data are means ± s.e.m. of the ratios of proBDNF optical intensity to the optical intensity of β-actin that serves to verify equal amounts of tissues. n = 5 (3 males and 2 females). **p < 0.05, *p < 0.01 compared to LMKR-treated in the same group. ##p < 0.05, #p < 0.01 compared to respective protein in the saline-treated group.

RETRACTED

In addition, we measured the tPA levels in both brain regions by Western blotting to confirm that the reduction in BDNF and proBDNF release in the prenatal cocaine-exposed brains was not caused by an alteration in tPA levels. The data summarized in (Fig 11) indicate that there were no discernible differences in tPA levels in the hippocampi [Basal: t(4) = 0.4055, p = 0.71230, K^+^: t(4) = 0.5769, p = 0.60443, NMDA/glycine: t(4) = 0.6767, p = 0.55359] and PFCX [t(4) = 0.80601, p = 0.46543, K^+^: t(4) = 0.7705, p = 0.48398, NMDA/glycine: t(4) = 0.7599, p = 0.48964] of prenatal cocaine- vs. saline-exposed rats.

**Fig 11:** Prenatal cocaine exposure did not alter the expression level of tPA in both hippocampi (a) and PFCX (b). The expression level of tPA in 50 μg post-mitochondrial (P2) fractions prepared from 10 μM NMDA/1 μM glycine or 65 mM K^+^ superfused hippocampal and PFCX slices of P21 prenatal cocaine- and saline-exposed rats were compared by Western blotting. Brain slices (100 μm x 100 μm x 3 mm) were superfused with 0.2 ml/min LMKR for 30 min or with 10 μM NMDA/1 μM glycine in LMKR for 10 min or 65 mM K+-depolarization for 1 min followed by 9 min with LMKR. Slices were collected, homogenized and centrifuged to obtain post-mitochondrial fractions. The blots were stripped and re-probed with anti-β-actin to validate equal loading. Densitometric quantification of blots revealed no discernible differences in tPA expression level. n = 4 (2 males and 2 females). Data are mean ± s.e.m. of the ratio of tPA to β-actin optical intensities.

## Discussion

We show here that prenatal cocaine exposure leads to adaptive hyperactivation of BDNF-TrkB signaling as indicated by heightened activated (pY) 145 KDa TrkB and increased NMDAR interaction with TrkB. These BDNF-induced TrkB signaling changes are caused by altered TrkB conformation and increased BDNF binding affinity resulting from dramatically reduced proBDNF and BDNF release at pre- and post-synaptic sites.

Prenatal cocaine exposure has profound deleterious effects on the function of dopamine D1 [8, 27–29], GABAergic [30] noradrenergic [31], AMPA [21], NMDA [30, 32] and mGluR1 [6, 33] systems. These findings suggest that prenatal cocaine exposure modifies synaptic plasticity and neurotransmission in multiple systems resulting in enduring brain function changes and cognitive impairments in later life [34, 35]. The functional alterations in prenatal cocaine-exposed brains are accompanied by structural changes including more synapses on synaptic spines [36], increased spine density [7] and elongated dendrites [8] in cortex and hippocampus, although reduced density and fewer cortical neurons have also been noted [37]. This discrepancy suggests that additional undefined molecular mechanisms contribute to the altered brain activities following *in utero* cocaine exposure.

RETRACTED

BDNF-TrkB signaling is essential for the tangential and radial neuronal migration in embryonic forebrain [38] and establishment of proper synaptic connectivity and brain function during the early postnatal period [39, 40]. BDNF-TrkB signaling regulates a complex range of neuronal activities, including cell survival, process outgrowth, neurotransmission, and synaptic plasticity to modulate cognition [41–43]. In support, intracerebroventricular administration of antisense BDNF oligonucleotides to maze-trained rats dampens their spatial memory [44], and maze-training itself increases activated TrkB levels in rodent hippocampi [45]. BDNF-induced TrkB activation engages NMDARs [23] to cause rapid NMDAR phosphorylation [46] and enhances glutamatergic neurotransmission [47] leading to LTP [43, 48]. The intimate interaction between BDNF-TrkB signaling and NMDAR function is further supported by *ex vivo* BDNF incubation of prenatal cocaine-exposed brains elevates both TrkB signaling and NMDAR-TrkB association. The increased BDNF-induced TrkB activation in the prenatal cocaine-exposed brains may therefore represent a neuroprotective adaptation in response to dampened NMDAR activity [32]. Similar increases in *ex vivo* BDNF-induced TrkB activation and signaling were observed in postmortem Alzheimer’s disease brains in which NMDAR function is severely compromised [49, 50]. BDNF-stimulated TrkB signaling activates ERK (pT^202^/pY^204^-ERK) and Akt (pS^473^-Akt) through the binding of adaptor proteins such as Shc and N-Shc to phosphotyrosine residues on activated TrkB [12]. Accordingly, the levels of Shc and N-Shc associated with activated TrkB following *ex vivo* BDNF incubation were higher in brains of prenatal cocaine-exposed P21 rats. While our data also show that *ex vivo* BDNF promotes tyrosine phosphorylation of the truncated form (95-KDa) of TrkB in both brain regions of P21 rats, prenatal cocaine has little effect on pY 95-KDa TrkB levels. The functional significance of the pY 95-KDa is however currently unknown.

Changes in BDNF-TrkB signaling during critical developmental stages greatly influence synaptic formation, brain architecture and function later in life [40]. Hence, the enhanced BDNF-TrkB signaling and TrkB-NMDAR interaction in prenatal cocaine-exposed brains may contribute to persistent cortical and sub-cortical structural and functional changes, including dendritic architecture and their synaptic connectivity [7, 8, 51] and neurotransmission particularly of glutamatergic systems [21, 30, 46–48]. As in our earlier report [23] showing that multi-day repetitive transcranial magnetic stimulation (rTMS) upregulates BDNF-TrkB signaling, we hypothesized that heightened BDNF affinity for TrkB is responsible for the enhanced BDNF response in prenatal cocaine-exposed brains. BDNF binds with two affinity states in prefrontal cortex and hippocampus, and prenatal cocaine exposure markedly increase both BDNF affinity states (Fig 7), as did the rTMS [23]. Presumably, BDNF binds with high-affinity (pM) to TrkB and low-affinity (nM) to p75^NTR^ [12]. The three-fold higher BDNF affinities in PFCX than in hippocampus imply subtle differences in BDNF interaction with TrkB and p75^NTR^ and the efficacies of TrkB/p75^NTR^ signaling in different brain regions. However, the BDNF concentration (50 ng/ml) used in the current *ex vivo* condition does not affect p75^NTR^ (Fig 3) and our separate studies indicate that prenatal cocaine exposure dampens p75^NTR^ function as demonstrated by the reduction in the p75^NTR^ and TRAF2/6 association in response to 200 ng/ml BDNF and proBDNF (data not shown). Since prenatal cocaine exposure did not result in discernible changes in TRAF2/6 and p75^NTR^, more thorough investigations are needed to elucidate the underlying mechanisms responsible for the reduced coupling of TRAF2/6 with p75^NTR^ in the prenatal cocaine exposed brains. Because the majority of full-length TrkBs in prenatal cocaine-exposed brains under non-stimulated conditions exhibited a higher *pI*, an altered TrkB conformation may underlie the observed higher affinity of BDNF for TrkB [52]. Alternatively, exposure to cocaine during gestation may also result in abnormal post-translational modifications such as glycosylation and phosphorylation of the TrkB that lead to conformational changes of this protein. Together, these results suggest that prenatal cocaine exposure elicits a conformational change in TrkB leading to a higher BDNF binding affinity to TrkB and more efficient BDNF-TrkB signaling that is accompanied by a defected p75^NTR^ system.

RETRACTED

To delineate the origin of TrkB conformational change and heightened BDNF binding affinity in prenatal cocaine-exposed brains, we determined the levels of activity-dependent BDNF and proBDNF release since overall proBDNF and BDNF expression was not altered. Prenatal cocaine exposure transiently reduces BDNF levels in embryonic forebrains early in gestation, which fully recover at later embryonic stages [38]. In our previous study, K^+^-depolarization and NMDA/glycine increased BDNF-TrkB signaling by promoting BDNF release, presumably from respective presynaptic neuronal terminals and postsynaptic dendritic fields [23]. We show here that K^+^-depolarization and NMDA/glycine elicit proBDNF and mBDNF release. More importantly, prenatal cocaine exposure profoundly reduced K^+^-depolarization and NMDA/glycine-evoked proBDNF and mBDNF release without affecting spontaneous pro-/m-BDNF efflux. Similarly, prenatal cocaine exposure reduces K^+^-induced BDNF release in hippocampus, cortex and striatum determined 1-week postnatally [53]. Thus, a reduced activity-dependent BDNF release in prenatal cocaine-exposed brains may lead to compensatory upregulation of BDNF-TrkB signaling to restore adequate synaptic activity.

ProBDNF may be converted into mBDNF intracellularly in the trans-Golgi by subtilisin-kexin of the endoprotease family such as furin, or in the immature secretory granules by proprotein convertases [54]. ProBDNF may also be secreted and converted to mBDNF via tPA-dependent activation of plasminogen and by matrix metalloproteases such as MMP[55]. BDNF and tPA have been implicated in the regulation of late-phase LTP (L-LTP) and long-term memory since mBDNF, but not the uncleavable proBDNF, rescues L-LTP in tPA and plasminogen knock-out mice [55]. These studies suggest that conversion of proBDNF to BDNF promotes L-LTP in the hippocampus and perhaps other brain regions. The dampened activity-dependent BDNF and proBDNF release without change in tPA level may indicate prenatal cocaine exposure negatively affects depolarization-exocytosis coupling and/or release of neurotransmitters and NMDAR function. Indeed, prenatal cocaine exposure reduces dopamine release [56] and NMDAR activity [32]. Altogether, these data demonstrate that prenatal cocaine exposure reduces pro-/m-BDNF release to upregulate BDNF-TrkB signaling and enhance TrkB-NMDAR coupling.

BDNF-TrkB signaling is linked to psychological distress and associated cognitive decline [50]. The functional Val66Met BDNF polymorphism that diminishes activity-dependent BDNF release predisposes an individual to depression, anxiety and cognitive impairment [57, 58]. In fact, prenatal cocaine-exposed mice heterozygous for the BDNF Val66Met cannot recall an extinguished cue-conditioned fear and have lower BDNF in medial prefrontal cortices immediately after this test [59]. Thus, reduced activity-dependent pro-/m-BDNF release, together with elevated BDNF-TrkB signaling un-opposed by a less effective p75^NTR^ following prenatal cocaine exposure may suggest that the offspring of pregnant cocaine users are more prone to depression, anxiety and certain cognitive impairments. In support of this depression/anxiety-prone hypothesis, exposure to relatively high doses of cocaine (40 mg/kg/day) and/or nicotine (5 mg/kg/day) *in utero* promotes depression and anxiety in aging rats [60]. Prenatal cocaine-exposed adolescent humans, however, exhibit impaired incidental face memory without changes in inhibitory control, working memory, and receptive language [61]. Moreover, prenatal cocaine exposure in humans causes subtle reductions in IQ and cognitive development [62, 63], delayed language development [64], and impaired performance in tasks requiring sustained attention [65]. Hence, the upregulated BDNF-TrkB signaling may either exacerbate synaptic damage [66] or be unable to fully adaptively offset the cocaine-elicited brain dysfunctions resulting in lesser capabilities to cope with psychological distress. Studies like ours help identify the molecular underpinnings to the prenatal cocaine-induced brain vulnerabilities and provide preventative therapeutic strategies to treat behavioral abnormalities. Importantly, the effects of prenatal cocaine exposure on brain function, synaptic activity and receptor functions assessed postnatally are similar whether cocaine was administered via intraperitoneal, subcutaneous or intravenous routes [6, 7, 8, 32, 33, 67], in different species [6, 7, 8, 33] or durations of treatment [6, 8, 30, 32, 33, 67]. Because a single intraperitoneal injection gives similar maternal and fetal plasma half-lives as in human studies [68], the current demonstration that the BDNF-TrkB system and its regulation are modified by intraperitoneal cocaine injection to pregnant rats suggests that similar effects could result from human *in utero* cocaine exposure.
